# Multiconstraint-Aware Routing Mechanism for Wireless Body Sensor Networks

**DOI:** 10.1155/2021/5560809

**Published:** 2021-03-31

**Authors:** Javed Iqbal Bangash, Abdul Waheed Khan, Asfandyar Khan, Atif Khan, M. Irfan Uddin, Qiaozhi Hua

**Affiliations:** ^1^Institute of Computer Sciences and IT, The University of Agriculture, Peshawar 25000, Pakistan; ^2^Department of IT and Computer Science, Pak-Austria Fachhochschule-Institute of Applied Sciences and Technology, Haripur, Pakistan; ^3^Department of Computer Science, Islamia College Peshawar, Peshawar, Pakistan; ^4^Institute of Computing, Kohat University of Science and Technology, Kohat 26000, Pakistan; ^5^Computer School, Hubei University of Arts and Science, Xiangyang 441000, China

## Abstract

The merger of wireless sensor technologies, pervasive computing, and biomedical engineering has resulted in the emergence of wireless body sensor network (WBSN). WBSNs assist human beings in various monitoring applications such as health-care, entertainment, rehabilitation systems, and sports. Life-critical health-care applications of WBSNs consider both reliability and delay as major Quality of Service (QoS) parameters. In addition to the common limitations and challenges of wireless sensor networks (WSNs), WBSNs pose distinct constraints due to the behavior and chemistry of the human body. The biomedical sensor nodes (BMSNs) adopt multihop communication while reporting the heterogeneous natured physiological parameters to the nearby base station also called local coordinator. Routing in WBSNs becomes a challenging job due to the necessary QoS considerations, overheated in-body BMSNs, and high and dynamic path loss. To the best of our knowledge, none of the existing routing protocols integrate the aforementioned issues in their designs. In this research work, a multiconstraint-aware routing mechanism (modular-based) is proposed which considers the QoS parameters, dynamic and high path loss, and the overheated nodes issue. Two types of network frameworks, with and without relay/forwarder nodes, are being used. The data packets containing physiological parameters of the human body are categorized into delay-constrained, reliability-constrained, critical (both delay- and reliability-constrained), and nonconstrained data packets. NS-2 is being used to carry out the simulations of the proposed mechanism. The simulation results reveal that the proposed mechanism has improved the QoS-aware routing for WBSNs by adopting the proposed multiconstraint-aware strategy.

## 1. Introduction

It can be observed from the history of human beings that getting older was an exception. Now, this trend is changing by the rapid increase in the elderly population living with chronic diseases and thus requires continuous monitoring [1]. According to the World Population Ageing 2019, the worldwide elderly population (65 + aged people) is expected to be increased from 703 million to 1500 million between 2019 and 2050 [2]. Similarly, according to the World Health Organization (WHO), the world's population of 60 + aged people between 2015 and 2050 will be almost doubled (12%–22%) [3]. The rate of growth in the elderly population is high in developing countries as compared to developed countries [4]. Besides the people suffering from chronic diseases, the patients inside the hospitals also require various levels of monitoring—ranging from a couple of times a day to continuous monitoring. The continuous and on-and-off health monitoring require a huge amount of additional medical and health-care costs [3]. WBSN has emerged to provide continuous and unsupervised physiological parameters monitoring of the human body. It may be helpful to solve the issues of chronic diseases, increased elderly population, and continuous and on-and-off in-hospital monitoring [5].

In WBSNs, the tiny, lightweight, cost-effective, and low-power BMSNs are implanted inside the human body to capture and observe the physiological parameters [6]. The heterogeneous nature of BMSNs generates various kinds of data packets that require different QoS parameters among which delay and reliability are of key importance [7]. There may be some data packets that require the shortest delay and highest possible reliability and others can allow some losses but need to assure the delivery with the shortest delay. Some data packets should be delivered with no or minimum losses but not within a specific time frame while others containing routine readings of physiological parameters do not have any such constraints.

The electromagnetic waves are absorbed by the human tissues during wireless communication among different in-body BMSNs as they are saline water in nature. The electromagnetic waves absorption and the energy consumed by the implanted BMSNs to carry out their routine operations are the two main reasons that may overheat the in-body BMSNs [8]. These overheated nodes may harm or affect the growth of human tissues [8]. Furthermore, in conventional wireless communication, path loss occurs due to two main reasons: multipath fading and free-space wave propagation. As WBSNs deal with the human body thereby resulting in high and dynamic path loss, therefore the conventional models used for path loss are not directly applicable. The reasons behind this dynamic and high path loss are the wireless communications among the different in-body BMSNs being through the human body and the human body movement [9].

The aforementioned issues of the WBSNs make routing a challenging task [10]. During the last decade, a number of routing protocols have been proposed to address the aforementioned issues that may be categorized based on QoS parameters, postural movement, and temperature rise. It is observed that most of the existing routing protocols are designed to address a single issue while few of them are designed to handle two of these issues. To the best of the authors' information, none of the existing routing protocols integrate the demanding QoS data, the human body movement, in-body wireless communications issues, and the overheating issue of the in-body BMSNs in their designs. In our previous research articles, critical data routing (CDR) [11] focuses on critical data, reliability aware routing (RAR) [12] considers reliability conscious data, and data-centric routing (DCR) [13] works on delay as well as reliability conscious data.

In this paper, the multiconstraint-aware routing mechanism is proposed which offers a more realistic solution that takes into consideration the various traits of the human body. It ensures the provision of the required QoS parameters by classifying the data packets into four categories: delay-constrained, reliability-constrained, critical, and nonconstrained. The routing decisions also incorporate the human body movement and in-body wireless communications issues. To mitigate the in-body overheating issue caused by antenna radiation absorption and energy consumption by nodes' circuitry, the routing mechanism takes into consideration the temperature rise of neighbor nodes during next-hop selection towards the body coordinator. It is a modular-based mechanism where various required tasks are performed by different modules.

The remainder of this paper is structured as follows: Section 2 presents the related literature of the existing routing mechanisms for WBSNs.  Section 3 provides the design and development details of the proposed routing mechanism. The performance assessment based on the simulation results of the proposed mechanism is discussed in Section 4. In the end, Section 5 concludes the paper and provides the possible future directions.

## 2. Related Literature

Due to the numerous applications of WBSNs, they have attained a tremendous focus of the research society. Recently the researchers have proposed various routing algorithms for WBSNs that might be categorized based on QoS parameters, postural movement, and temperature rise. It is observed that most of the existing routing protocols are designed to address a single issue while a few of them are designed to handle two of these issues. The captured physiological parameters demand different QoS parameters and can be classified as critical data (CD), reliability-conscious data (RCD), delay-conscious data (DCD), and nonconscious data (NCD) [7,13–15]. QPRD [14] uses RCD and NCD and QPRR [15] uses DCD and NCD, while ZEQoS [16] uses DCD, RCD, and NCD classes of data. All these routing schemes are designed considering a hospital-based scenario where the physiological parameters are displayed. PARA [17] classifies the captured data into emergency, on-demand, and periodic classes. All these routing schemes take care of the demanding QoS parameter and are not considering the overheated nodes and human body movement issues of WBSNs. The routing mechanisms considering the demanding QoS data have shortcomings in their decision making while selecting a suitable next hop. Some of them such as QPRD, QPRR, and ZEQoS consider the demanding QoS parameter on the node level. Others such as TQMoS use a minimum hop-count strategy in the selection of suitable next hop for all types of data; even the RCD packets can tolerate some delays. Secondly, it uses redundant transmission for CD packets.

Both TMQoS [7] and TLQoS [18] categorize the captured data into four classes and also try to minimize the temperature rise of the in-body BMSNs by avoiding the overheated nodes as forwarder nodes. All the aforementioned QoS-based routing protocols are based on modular approach where every task is performed using a separate module. Besides the demanding QoS, these schemes also take care of the energy consumption being one of the important issues. TMQoS and TLQoS consider both the demanding QoS and overheated nodes issue but overlook the human body movement.

TARA [19], being the first routing protocol of WBSNs addressing the overheated nodes issue, looks at the activities of the neighbors to evaluate the level of the temperature rise. It is based on the withdrawn policy to forward the data using nonoverheated nodes. LTR [20] is another routing scheme where the next-hop selection decision is made by not considering the overheated nodes. On the other hand, LTRT [21] based on Dijkstra's algorithm evaluates the end-to-end path temperature level and follows the path having less temperature level. The routing protocols addressing the overheated nodes issue overlook the demanding QoS of the captured data and human body movement. TTRP [22] is another routing protocol that considers the trust and overheated nodes while selecting the next-hop node. MTR [23] is the only routing protocol that considers both the overheated nodes issue along with the human body movement but it overlooks the high path loss due to the in-body wireless communication and demanding QoS data.

ATEAR [24] is a temperature- and energy-aware routing scheme that uses a block-chain to reduce the temperature rise and energy consumption. CEPRAN [25] uses a cooperative approach for communication to enhance energy efficiency and reliable communication. EHCRP [26] consider several parameters for routing decisions to achieve the desired goal, i.e., energy efficiency. Similarly, the authors in [27] also aim to efficiently use the energy of the sensor nodes, while [28] aims to do the same but considers only critical data (CD).

To cope with the human body movement, different routing protocols such as [9,29–32] have been proposed. All these routing protocols consider the human body movement and its effects. Furthermore, most of them have also worked on energy efficiency being among the key issues of WBSNs. All of them overlooked the demanding QoS data and overheated nodes issue. Moreover, they are also not considering the high path loss due to in-body wireless communication. It is the main reason that the normal path loss models cannot be used with WBSNs. Authors in [33–35] have another interesting concept of using relay nodes along with BMSNs. The BMSNs are used only to capture the required physiological parameters and send them to the nearby relay node while the relay/forwarder nodes are used to forward the received data. Some researchers have used the relay/forwarder nodes to utilize the energy of the BMSNs efficiently while others have used it to address the path loss issue.

To the best of our information, none of the existing routing protocols integrate the demanding QoS data, human body movement, high path loss due to in-body wireless communication, and the overheating issue of the in-body BMSNs in their designs. In our previous research articles, critical data routing (CDR) [11] focuses on critical data, reliability aware routing (RAR) [12] considers reliability conscious data, and data-centric routing (CDR) [13] works on both delay- and reliability-conscious data. All these schemes also consider the human body movement, high path loss due to in-body wireless communication, and the overheating nodes issue.

### 2.1. Proposed Mechanism

The aforementioned research gap is addressed by the proposed routing mechanism, which considers the demanding QoS data, overheating nodes, human body movement, and wireless communication through the human body.

### 2.2. Network Frameworks

Two types of network frameworks, with and without relay/forwarder nodes, are being used in the proposed routing mechanism, which is discussed as follows.

Multiconstraint-aware routing mechanism without relay/forwarder nodes (MCARM): the scanned images are in this type of network framework as shown in Figure 1; different in-body BMSNs and on-body local coordinator (LC) can be grouped together using graph theory as in [13]

(1) $$\begin{array}{c} G=\left(V,E_{d}\right), \end{array}$$

where V is the combination of both S and LC as in (2) [13] and S is the set of N in-body BMSNs as in (3) [13]:

(2) $$\begin{array}{c} V=\left\{S\right\}U\left\{LC\right\}, \end{array}$$

(3) $$\begin{array}{c} S=\left\{s_{1},s_{2},s_{3},\ldots ,s_{n}\right\}. \end{array}$$

Similarly, Ed denotes the set of *M* possible in-body wireless communication connections, connecting two BMSNs or a BMSN and LC as in [14]

(4) $$\begin{array}{c} E_{d}=\left\{e_{1},e_{2},e_{3},\ldots ,e_{m}\right\}. \end{array}$$

Multiconstraint-aware routing mechanism with relay/forwarder nodes (MCARMR): in this type of network framework as shown in Figure 2, the job of the BMSNs is to capture only the physiological parameters of the human body while they are forwarded using a different type of nodes called relay/forwarder nodes. The concept of the relay/forwarder nodes is already being used in [33–35].

This type of network framework can be modeled as in (1). V is the combination of S, RN, and LC as in (5) [13]. Similarly, Ed denotes the set of *M* possible wireless connections, connecting two relay/forwarder nodes, or a relay/forwarder node, and a BMSN same as in (4).

(5) $$\begin{array}{c} V=\left\{S\right\}U\left\{RN\right\}U\left\{LC\right\}. \end{array}$$

S is the set of N in-body BMSNs same as in (3) and RN is the set of *M* wearable relay nodes as in [13]

(6) $$\begin{array}{c} RN=\left\{r_{1},r_{2},r_{3},\ldots ,r_{m}\right\}. \end{array}$$

### 2.3. Classification of Captured Data

The captured data packets containing the physiological parameters of the human body are different in terms of the demanding QoS parameters. In this research work, the data packets are classified into four different categories same as in [7,13–15]. These four types of data packets, shown in Figure 3, are discussed below.

#### 2.3.1. Nonconscious Data (NCD)

This type of data packet reflects the normal and routine reading and does not enforce any time-deadline and/or reliability constraint. Body temperature, blood pressure, heartbeat, etc. are the examples of NCD packets.

#### 2.3.2. Delay-Conscious Data (DCD)

This type of data packets is time-critical imposing delay constraint and reasonable packet losses are acceptable. Video imaging, telemedicine, EMG, and motion sensing are examples of DCD packets.

#### 2.3.3. Reliability-Conscious Data (RCD)

This type of data packet needs to be transmitted with minimum or no packet losses and can tolerate some delays. Respiration monitoring and pH-level are examples of RCD packets.

#### 2.3.4. Critical Data (CD)

This type of data packet is the most important and reflects the life-critical physiological parameters of the patients. The critical data (CD) packets impose strict delay as well as reliability constraints. This type of data packet is the most important and reflect the life-critical physiological parameters of the patients. The CD packets impose strict constraints in terms of both delay and reliability. ECG and EEG monitoring in a critical situation such as medical surgery, brain stroke, and heart attack, and other physiological parameters that indicate the critical value require real-time and reliable monitoring.

## 3. Proposed Multiconstraint-Aware Routing Mechanism

This section discusses the proposed routing mechanism that considers the demanding QoS data, overheated nodes, human body movements, and in-body wireless communication. It ensures selecting the best suitable route based on the data packet types by considering end-to-end delay and reliability. It takes care of the high path loss due to in-body wireless communication and dynamic path loss caused by human body movement and tries to avoid the overheated nodes while deciding the next-hop node. It is a cross-layer modular approach, where each module is assigned its duty.

The block diagram shown in Figure 4 consists of Packets Divider (PD), Data Packets Divider (DPD), MAC Receiver (MAC-R), Delay Calculator (DC), Reliability Calculator (RC), Link Quality Calculator (LQC), Temperature Calculator (TC), Routing Unit (RU), QoS-Conscious Next-Hop Selector (QoS-CNHS), QoS-Conscious Queues (QoS-CQs), and MAC Transmitter (MAC-T). The packets either Hello Packets (HPs) or Data Packets (DPs) transmitted by the neighborhood node or LC are received at MAC-R, and it is the job of the PD to divide the Hello and Data Packets using Algorithm 1. The HPs are forwarded towards RU while DPs are forwarded towards DPD. Similarly, it is the job of the MAC-T to transmit the HPs as well as DPs (either generated or received) towards the neighborhood nodes and/or LC. The DPs received from PC, and the DPD has to divide them as critical data (CD), reliability-conscious data (RCD), delay-conscious data (DCD), and nonconscious data (NCD) using Algorithm 2 and forward them towards QoS-ANHS. The other units of the proposed routing mechanism are discussed as follows.

### 3.1. Delay Calculator (LC)

At each node Ni, it is the job of the DC to calculate the Node Delay NDNi using (7) [13]. QDNi is the delay that occurred in queue and TLi,j is the delay that occurred during transmission of the DPs from Ni to Nj using Wireless Link WLi,j. The other types of delays, i.e., propagation and processing, are small enough to be ignored.

(7) $$\begin{array}{c} ND_{Ni}=QD_{Ni}+TD_{ij}, \end{array}$$

where QDNi given in (8) [36] is the time that a DP spends in waiting for transmission, where *α*, the constant factor value, ranges from zero to one and in most cases such as [7,13,14,16] it is equal to 0.2. The queue delay QDNi occurred once the first delay-conscious or critical data packet is transmitted.

(8) $$\begin{array}{c} QL_{Ni}=\alpha QL_{Ni}+\left(1-\alpha \right)QL_{Ni}. \end{array}$$

TLi,j given in (9) [16] is the time that a DP spends in waiting at the MAC layer, where NP represents the number of DPs transmitted, DRbits is the generated data rate (bits), and SPbits is the packet size (bits).

(9) $$\begin{array}{c} TL_{i,j}=\left(\frac{1}{DR_{\text{bits}}}\right)x\left(\frac{\sum_{z=1}^{NP}SP_{\text{bits}}\left(Z\right)}{NP}\right). \end{array}$$

### 3.2. Reliability Calculator (RC)

RC is used to calculate the reliability of wireless link WLi,j denoted by LRi,j from Ni to Nj using (10) [37]. *β* represents the weighting factor with values from zero to one and *ß* equal to 0.4 is being used to simulate the proposed routing mechanism same as in [6,10–12,14,15] and Pave is given in (11) [13], where NPsucc is the number of successfully transmitted packets and NPtotal represents the total transmitted packets.

(10) $$\begin{array}{c} LR_{i,j}=\beta LR_{i,j}+\left(1-\beta \right)\times P_{\text{ave}}, \end{array}$$

(11) $$\begin{array}{c} P_{\text{ave}}=\frac{NP_{\text{succ}}}{NP_{\text{total}}}. \end{array}$$

### 3.3. Link Quality Calculator (LQC)

The job of LQC is to calculate the quality of wireless link WLi,j represented by WLQi,j from Ni to Nj. Equation (12) [38] is being used which is based on a semiempirical formula to calculate the path loss PLi,j in terms of the distance di,j (the distance of Ni from Nj). The path loss exponent is denoted by *n* and PL0 is the reference link quality at distance d0.

(12) $$\begin{array}{c} PL_{i,j}=PL_{0}+10n\;\log\frac{d_{i,j}}{d_{0}}. \end{array}$$

To accommodate the dynamic human body movements, “Zero-Mean Gaussian Random Variable X∂ having Standard Deviation ∂” is being used to formulate (13) [13] from

(13) $$\begin{array}{c} PL_{i,j}=PL_{0}+10n\;\log\frac{d_{i,j}}{d_{0}}-X_{\partial }. \end{array}$$

Equation (14) is to calculate the link quality WLQi,j of wireless link WLi,j from Ni to Nj can be calculated using (14) [38] derived from (13), where Ptrans is the transmission power and WLQthre represents the threshold level of the link quality.

(14) $$\begin{array}{c} WLQ_{i,j}=\frac{1}{2}-\frac{1}{2}\text{erf}\left(\frac{-P_{\text{trans}}+PL_{i,j}+WLQ_{\text{thre}}}{\sqrt{2\pi \partial }}\right). \end{array}$$

### 3.4. Temperature Calculator (TC)

The task assigned to TC is to calculate the increase in the temperature of any in-body BMSN Ni. The rate at which the electromagnetic waves are absorbed by the human tissues during wireless communication, known as specific absorption rate (SAR), is given in (15) [19], where *σ* refers to the electric conductivity, the induced electric field is represented by *E*, and the density is denoted by *ρ*.

(15) $$\begin{array}{c} \text{SAR}=\frac{\sigma \left|E\right|2}{\rho }. \end{array}$$

Similarly, the in-body BMSNs consume energy to perform the various tasks, which is the second reason that causes an increase in their temperature. Pennes Bioheat formula [39] given in (16) can be used to measure the rate of temperature increase dT/dt due to energy consumption, where the temperature increase (TI) due to thermal conductivity is denoted by K∆2T, b(T – Tb) refers to TI caused by blood perfusion, *ρ*SAR represents the TI due to electromagnetic waves absorption, Pc is the TI due to energy consumption of the BMSNs' circuitry, *ρ* refers to the mass density, and Cp represents the specific heat of the human tissue. The aforementioned parameters of (16) are assigned the values provided by [35]

(16) $$\begin{array}{c} \frac{dT}{dt}=\frac{K\Delta^{2}T-b\left(T-T_{b}\right)+\rho SAR+P_{c}}{\rho C_{p}}. \end{array}$$

### 3.5. Routing Unit (RU)

RU is further divided into three subunits, namely, Routing Table (RT), Routing Table Constructor (RTC), and Hello Packets Generator (HPG). The job of RTC is to create and/or update the RT periodically using the data provided by various parameter calculators and neighborhood nodes through Hello Packets (HPs). Once an HP is received from a neighborhood node Nj, the node Ni compared the temperature increase TINj to a predefined level known as Temperature Increase Threshold TIthre. The RT is not updated and the HP is dropped if the TINj ≥ TIthre and the entry of Nj are removed from the RT if any. Based on the received data, path delay PDi, j, LC, path reliability PRi, j, LC, and path temperature PTi, j, LC from source Ni to the destination (LC) through Nj are calculated using (17)–(19) same as in [13], respectively.

(17) $$\begin{array}{c} PD_{i,j,LC}=PD_{i,j,LC}+ND_{Ni}, \end{array}$$

(18) $$\begin{array}{c} PR_{i,j,LC}=PR_{i,j,LC}+NR_{Ni}, \end{array}$$

(19) $$\begin{array}{c} PT_{i,j,LC}=PT_{i,j,LC}+TI_{Nj}. \end{array}$$

Figure 5 shows the organization of RT for the proposed routing mechanism, containing destination (LC) address and location, neighborhood node Nj address and location, wireless link quality WLQi, j (between Ni and Nj), path (from Ni to LC using Nj as next-hop) delay, path (from Ni to LC using Nj as next-hop) reliability, and path (from Ni to LC using Nj as next-hop) temperature.

Once the RT is created and/or updated periodically, Hello Packet Generator (HPG) is responsible for constructing the HP based on the available information. The HP is forwarded towards MAC-transmitter which broadcasts it among the neighborhood nodes.

### 3.6. QoS-Conscious Next Hop Selector (QoS-CNHS)

The responsibility of the QoS-CNHS is to choose the suitable next-hop as required by the demanding QoS data packets. Once the DPs are classified as CD, DCD, RCD, and NCD packets in Data Packets Divider (DPD), the proposed Algorithm 1 for QoS-CNHS examines the RT and neighbor nodes (NNs) having WLQi,*j* ≥ WLQthre are selected among all neighborhood nodes and placed in NHNWLQ (Next-Hop Neighbors with acceptable wireless link quality) (lines 3–5). If NHNWLQ is empty, then the DP is dropped (lines 8–9). If it is not empty, then DP is examined for its type. In case the DP is either CD or DCD packet, then DP and NHNWLQ are sent to the delay-conscious procedure (lines 10–11). If DP is RCD packet, then DP and NHNWLQ are sent to the reliability-conscious procedure (lines 12–13). Suitable Next-Hop (SNH) is the NN with minimum PTi,j, LC in NHNWLQ for NCD packet, and the DP is forwarded to the NCQ (lines 14–16).

The delay-conscious procedure is responsible for the CD and DCD packets and after receiving DP and NHNWLQ, it looks at NHNWLQ, and NNs with PDi,j, LC ≤ PDthre are listed into NHNPD (Next-Hop Neighbors with acceptable path delay) (lines 19–22). DP is dropped if NHNPD is empty (lines 23-24) and if there is only one NN in NHNPD, then it is selected as SNH (lines 25-26). DP is sent towards DCQ if it is DCD packets (lines 27-28); otherwise it is sent towards CDQ (lines 29–31). In case of more than one NN in NHNPD, then the NN with minimum PTi,j, LC is selected as SNH for DCD packet and DP is sent towards DCQ (lines 32–34), while DP and NHNPD are sent to the reliability-conscious procedure for CD packet (35-36).

The reliability-conscious procedure is called for CD and RCD packets and after receiving DP and NHNWLQ or NHNPD, it looks at the received list, and NNs with PRi,j, LC ≥ PRthre are recorded into NHNPR (Next-Hop Neighbors with acceptable path reliability) (lines 39–42). SNH is the NN with the highest PRi,j, LC if NHNPR is empty (lines 43–45) and RCD packet is sent towards RCQ (lines 46-47) while CD packet is sent towards CDQ (lines 48–39). In case of having only one NN in NHNPR, it is selected as SNH (lines 50-51) and RCD packet is sent towards RCQ (lines 52-53) while CD packet towards CDQ (lines 53–56). In case of more than one NNs in NHNPR then NN with minimum PTi,j, LC is selected as SNH (lines 57-58). RCD packet is sent towards RCQ (lines 59-60) while CD packet is sent towards CDQ (lines 61-62). Flowchart for the proposed QoS-CNHS algorithm is given in Figure 6.

QoS-Conscious Queues (QoS-CQs): after selecting the suitable next-hop node as required by the demanding QoS data packets, they are forwarded towards QoS-CQs. Four types of QoS-CQs are being used, where Critical Data Queue (CDQ) is at the highest priority, next is Delay-Conscious Queue (DCQ), then comes Reliability-Conscious Queue (RCQ), and finally Nonconscious Queue (NCQ) is having the lowest priority. The CD packets are placed in CDQ while DCD packets are placed in DCQ until the MAC-transmitter sends them towards the selected next-hop. Similarly, the RCD and NCD packets are retained in RCQ and NCQ before being transmitted by the MAC-transmitter, respectively. To cope with indefinite waiting, the data packets in low-priority queues are moved into the high-priority queues same as in [7,11–16].

### 3.7. Simulation and Performance Assessment

In this section, the simulation of the proposed routing mechanism is discussed along with its performance assessment against other related and recent mechanisms.

### 3.8. Simulation Setup

Network Simulator version 2 (NS2) [35] is used to carry out the simulation and performance evaluation of the proposed routing mechanism for WBSNs same as in [11–13]. It is an open-source, event-driven discrete-time simulator, which is designed to facilitate the research activities of networking and communication. It supports simulating TCP, multihop routing, and multicasting algorithms by having complete models for physical, data-link, and MAC layers.

Two types of network frameworks with and without relay/forwarder nodes (RNs) denoted as MCARM and MCARMR, discussed in Section 3.1, are being used in order to assess the performance of the proposed mechanism with other recent and related mechanisms. Some of the BMSNs are used to generate conscious (either RCD, DCD, or CD) packets and others nonconscious (NCD) packets. The proposed mechanism is implemented in such a way that every BMSN is used to generate all types of data packets discussed in Section 3.2 to get the average results. The performance of the proposed mechanism is assessed against TQMoS [6] and LTRT [20]. TQMoS considers both the demanding QoS data and the temperature increase of the in-body BMSNs. Similarly, LTRT is designed to address the temperature increase issue that uses path temperature while selecting the next-hop node. The proposed mechanism is assessed in terms of average on-time packet delivery ratio for CD and DCD packets, packet loss ratio due to in-body wireless communication and human body movements (path loss), average end-to-end-delay for DCD packets, average packet delivery ratio for CD and RCD packets, maximum temperature increase, and average energy consumed. The simulation results reveal that the proposed mechanism has improved the QoS-aware routing for WBSNs by adopting a multiconstraint-aware strategy. The network parameters used in simulating the proposed routing mechanism for WBSNs are as in Table 1.

## 4. Simulation Results and Discussion

The performance evaluation of the proposed MCARM and MCARMR against other mechanisms in terms of the aforementioned parameters is shown and discussed in the following sections.

### 4.1. Packet Loss Ratio (PLR)

The average PLR against wireless link qualities (WLQs) considering different data generation rates by averaging the results is given in Figure 7. It shows that the PLR is high at a very tight WLQ level for TQMoS, LTRT, and MCARM and is decreasing as its threshold level is becoming low. However, it remains almost consistent for MCARMR at different WLQ [40] threshold levels. Moreover, MCARM results in slightly poor performance compared to MCARMR [41] and significantly good performance when compared with TQMoS and LTRT. TQMoS and LTRT are not considering the in-body wireless communication and human body movements, which are the reasons for their low performance. Furthermore, TQMoS performs well when compared with LTRT because of the provision of the demanding QoS data.

### 4.2. Average Packet Delivery Ratio (APDR)

In this section, the performance of both MCARM and MCARMR is assessed considering both the reliability-conscious and critical data in terms of APDR.

### 4.3. Reliability-Conscious Data (RCD)

Figure 8 illustrates the APDR of RCD packets against data generation rates (DGRs) at different wireless link qualities by averaging their results. It is observed from the figure that for mechanisms the APDR is slightly reducing as the DGR is growing high which is due to the increased network congestion. The figure shows that, at high DGR, MCARM performs well when compared with all three but at medium and low DGRs it is replaced by MCARMR [42]. The reason is the increased traffic congestion on the RNs at high DGR. Furthermore, it is also observed that TQMoS shows better results when compared with LTRT at all DGRs.

TQMoS considers the temperature increase issue of the in-body BMSNs along with the provision of the demanding QoS data but completely ignores in-body wireless communication and human body movements issues. Secondly, it uses a minimum hop-count strategy while selecting the suitable next-hop; even RCD packets can tolerate some delays. Similarly, the aim of LTRT is to address the temperature increase issue of in-body BMSNs and completely overlooks the in-body wireless communication and human body movement's issues along with the provision of the demanding QoS data.

### 4.4. Critical Data (CD)

The APDR of the critical data (CD) packets is given against DGRs at different wireless link qualities by taking an average of their results in Figure 9. By comparing Figures 8 and 9, it is observed that the performances of MCARM and MCARMR are almost the same for both RCD and CD packets in terms of APDR for all DGRs. TQMoS results in a slightly low packet delivery ratio at low DGR but with the increase in the DGRs, its performance is becoming poorer in CD packets compared to RCD packets. It uses redundant transmission of CD packets [42], causing high network congestion which results in comparatively low APDR. Furthermore, there is no effect on the performance of LTRT as it does not consider the provision of the demanding QoS data.

### 4.5. Average End-to-End Delay (AEED)

Figure 10 shows the AEED of the delay-conscious data (DCD) packets against different DGRs at various wireless link quality threshold levels by averaging their results. The figure illustrates that the TQMoS performs slightly better than MCARM, MCARMR, and LTRT because the suitable next-hop selection procedure of TQMoS uses hop-counts. MCARM results in slightly high AEED as compared to TQMoS but outperforms the MCARMR and LTRT. In both MCARM and MCARMR, the selection of suitable next-hop is based on the path delay and wireless link quality level for DCD packets [43]. Furthermore, LTRT results in high AEED among all due to its ignorance about the provision of the demanding QoS data.

### 4.6. On-Time Average Packets Success Ratio (OTAPSR)

This section presents the performance assessments of both MCARM and MCARMR in terms of OTAPSR for delay-conscious data (DCD) and critical data (CD) packets.

### 4.7. Delay-Conscious Data (DCD)

The OTAPSR of DCD packets against demanded Time-To-Leave (TTL) deadline and considering different wireless link quality threshold levels by taking the average of their results at high and low DGR is shown in Figures 11(a) and 11(b), respectively. The figures clarify that MCARM performs well when compared with other mechanisms considering both high and low DGRs at very tight TTL deadlines. As the TTL deadline is becoming relaxed, MCARMR results in improved performance when compared with others at low DGR. For high DGR, its performance remains below MCARM because of high network congestion on the RNs caused by high DGR [44]. At tight TTL deadlines, the slightly poor performance of MCARMR compared with MCARM considering both high and low DGRs is because of the delays at the RNs.

The performance of TMQoS and LTRT in terms of OTAPSR for DCD packets is improving as the TTL deadline becomes relaxed; however, they are still poorly performing when compared to MCARM and MCARMR due to not considering the in-body wireless communication and human body movements. TQMoS results in improved performance compared to LTRT because of the provision of demanding QoS data which is not considered by LTRT.

### 4.8. Critical Data (CD)

Figures 12(a) and 12(b) illustrate the OTAPSR for CD packets against demanded TTL at different wireless link quality threshold levels by averaging their results at high and low GDGRs, respectively. By comparing the results of TQMoS for DCD packets with CD packets, it is clear that it gives comparatively better results for DCD packets because of the redundant transmission in the case of the CD packets. Moreover, there is no difference in the results of other mechanisms.

### 4.9. Maximum Temperature Increase

Figures 13(a) and 13(b) present the maximum temperature increase of the in-body BMSNs for DCD/RCD/NCD packets and CD packets against DGRs at different wireless link quality threshold levels by averaging their results, respectively. It is clear that the temperature increase is becoming more with the rise in the DGRs for all mechanisms. More communications occur at high DGR that results in a temperature increase of the in-body BMSNs [45]. MCARMR results in a lower temperature increase when compared with other mechanisms because the RNs are used to forward the captured data of the BMSNs. LTRT outperforms MCARM and TQMoS as its main aim is to address the temperature increase issue of the in-body BMSNs.

In the case of DCD/RCD/NCD packets, TQMoS is poorly performing as compared to MCARM because of its minimum hop-count based on suitable next-hop selection strategy. Furthermore, by comparing the maximum temperature for TQMoS in the case of DCD/RCD/NCD packets and CD packets, it is observed that it results in more temperature increase in the case of CD packets when compared with DCD/RCD/NCD packets. This is because of the redundant transmission of CD packets resulting in more communication and more communication means high temperature increase. The results of LTRT, MCARM, and MCARMR remain the same considering both DCD/RCD/NCD packets and CD packets.

### 4.10. Average Energy Consumption (AEC)

The AEC of the in-body BMSNs for DCD/RCD/NCD packets and CD packets against DGRs at different wireless link quality threshold levels by taking the average of their results is shown in Figures 14(a) and 14(b), respectively. It is clear that the increase in DGRs increases the AEC in both cases for all mechanisms. The high energy consumption is due to more communication caused by high DGR. It is observed that MCARMR outperforms the others as the BMSNs are not involved in communicating the data of other BMSNs which consumes more energy among all tasks performed by the sensor node. LTRT consumes more energy when compared with other mechanisms because of its main aim of addressing the temperature increase issue and not considering the energy consumption. TQMoS is poorly performing in the case of CD packets when compared to MCARM because of the redundant transmission of CD packets. On the other hand, TMQoS shows improved performance when compared with MCARM because of its minimum hop-count suitable next-hop selection strategy.

## 5. Conclusion and Future Directions

WBSN is the medical and health-care application of WSNs offering continuous remote monitoring of different vital-signs information of the human body. Along with inherited limitations and challenges of WSNs, WBSNs pose distinct constraints due to the behavior and chemistry of the human body. The diversity of the generated data from BMSNs demands different QoS parameters in the delivery of the data to the local coordinator (LC). In addition to the demanding QoS data, the routing mechanisms need to be aware of the temperature increase of in-body BMSNs, in-body wireless communication, and human body movement issues. The existing routing mechanisms in this domain have partially addressed these issues. This research work has integrated the aforementioned issues by adopting a multiconstraint-aware strategy. Two types of network frameworks with and without relay/forwarder nodes are being used. The data packets containing physiological parameters of the human body are categorized into delay-constrained, reliability-constrained, critical (both delay- and reliability-constrained), and nonconstrained data packets. The proposed routing mechanism offers a more realistic solution with the dynamics of the human body. The contributions of the proposed routing mechanism have demonstrated better results in terms of latency, reliability, temperature increase, and energy efficiency when compared with the existing work.

The possible future directions could be the integration of the proposed mechanism with inter-WBSNs, ensuring the privacy of the patients' vital-signs information, the optimal number of RNs and their placement, prolonging networks' lifetime, and assessment using test-bed through real-world implementation.

## Figures and Tables

**Figure 1:** Network framework without relay/forwarder nodes.

**Figure 2:** Network framework relay/forwarder nodes.

**Figure 3:** Classification of captured data.

**Figure 4:** Block diagram of proposed multiconstraint-aware routing mechanism.

**Figure 5:** Routing table organization of the proposed routing mechanism.

**Figure 6:** Flowchart of the proposed QoS-CNHS algorithm.

**Figure 7:** Average PLR vs. WLQ thresholds at different DGRs.

**Figure 8:** APDR vs. DGRs at different WLQs for RCD packets.

**Figure 9:** APDR vs. DGRs at different WLQs thresholds for CD packets.

**Figure 10:** AEED vs. DGRs at different WLQ thresholds for DCD packets.

**Figure 11:** OTAPSR vs. required TTL deadlines for DCD packets at (a) high DGR and (b) low DGR.

**Figure 12:** OTAPSR vs. required TTL deadlines for CD packets at (a) high DGR and (b) low DGR.

**Figure 13:** Maximum temperature increase of BMSNs vs. DGRs for (a) DCD/RCD/NCD and (b) CD packets.

**Figure 14:** AEC of BMSNs vs. DGRs for (a) DCD/RCD/NCD and (b) CD packets.

**Algorithm 1:** QoS-conscious next-hop selector algorithm.

**Table 1:** Network parameters used in simulation.

Parameters	Value
Nodes quantity (MCARM)	14 (BMSNs) + 1 (LC)
Nodes quantity (MCARMR)	14 (BMSNs) + 14 (RNs) + 1 (LC)
Communication range (MCARM)	40 cm
Communication range (MCARMR)	20 cm (BMSNs) and 40 cm (RNs)
Initial energy	100 joules
Bit error rate (BER)	10^−2^ – 10^−4^
Communication power (MCARM)	8.5872e^−4^
Communication power (MCARMR)	8.5872e^−4^ (BMSNs) and 1.0872e^−4^ (RNs)
Propagation model	TwoRayGround
Buffer size	60 packets
Application type	Event-driven
Type of traffic	Constant bit rate (CBR)
MAC layer protocol	IEEE 802.15.4
Type of network interface	WirelessPhy
Simulation time	1000 seconds

## Data Availability

The data used to support the findings of this study are included within the article (see Table 1).
